# Analysis of Legal Attributes and Rights Attributes of Personal Information from the Perspective of Big Data

**DOI:** 10.1155/2022/9731414

**Published:** 2022-06-17

**Authors:** Jingzhong Yan

**Affiliations:** ^1^Kenneth Wang School of Law, Soochow University, Suzhou, Jiangsu 215007, China; ^2^Business School, Suqian University, Suqian, Jiangsu 223800, China

## Abstract

With the popularization and rapid development of Internet technology (IT), social activities based on the exchange of personal information are rapidly popularizing. Although the free flow of a huge volume of personal data meets the needs of information exchange, its illicit use poses legal risks to rights holders and infringes on the applicable rights and interests of the information subject. The ambiguity of the right attribute and legal attribute of personal information leads to the scattered protection of personal information in the legislative system in different legal norms. Based on this background, this paper constructs an evaluation index based on the legal attributes and rights attributes of personal information rights and proposes a rationality evaluation method for the attributes of personal information rights based on neural networks. The completed work is as follows: (1) focusing on the legal attributes and the right attribute is discussed in detail, and the dissimilar views of scholars at home and abroad are presented. (2) The back propagation neural network (BPNN) model structure required in this study is defined, and the evaluation index based on the legal attribute and right attribute of personal information right is produced. (3) Use big data technology to collect relevant data and compare the results obtained by the BPNN model with the results obtained by the improved BPNN model. The results show that the improved BPNN evaluate model has smaller error and higher accuracy.

## 1. Introduction

With the development of the Internet, more and more attention has been paid to the protection of personal information, which is closely related to the characteristics of the relevant subjects, and can accurately identify the identity of the information subject, thus reflecting the particularity of the subject in society, including the identity of the individual, family, property status, and medical health. Article 111 of the “General Principles of Civil Law” has formulated a special law for the protection of personal information. This article clarifies the relevant guidelines that others should follow when using citizens' information [1]. In the information age, this is the era's necessity for the security of personal information, and it expresses society's intent. The legislative spirit of this article is to affirm that personal information is a private interest enjoyed by natural persons in accordance with the law, and such private interests are protected by legal coercive force, which also ensures the freedom of natural persons to exercise personal rights within a certain range. At the same time, the right to personal information has the attribute of willpower. In this regard, the right to personal information should belong to a civil right, not a general legal interest. First of all, the right to personal information protects the specific interests of natural persons and is a collection of natural persons' spiritual interests and property interests. The “General Principles of Civil Law” provides legal protection for such specific interests [2]. Personal information encapsulates the private interests of natural persons; therefore, the subject of personal information should be safeguarded under the right to personal information. This kind of private interest is mainly reflected in two aspects: on the one hand, when personal information is infringed by others, the natural person can request the relevant authorities to protect it, and at the same time, it can also require the relevant infringer to act or refrain from taking certain actions, so that the right holder can independently decide how your personal information will be used. This not only reflects the freedom of civil subjects to exercise relief methods when they are violated but also demonstrates the personal dignity and personal interests of civil subjects but also shows the protection of civil subjects by laws and regulations, and it is guaranteed that civil subjects can realize their relevant legal interests of personality in civil activities. On the other hand, the law allows the right holder to freely dominate and control personal information within a certain range, which is mainly manifested in the commercial use of the personal information by the right holder, and in the process realizes a certain property value of the personal information, which reflects the freedom of civil subjects to exercise civil rights [3]. Secondly, the right to personal information has the attribute of willpower, and the essential attribute of civil rights is the willpower, which is the right granted by the law to civil subjects to make independent decisions within a specific range. This attribute of willpower is the fundamental characteristic of civil rights, and it is also the fundamental characteristic that distinguishes civil rights from general legal interests [4]. For example, in the theory of ownership, the right holder can independently control and dominate the property and exclude the interference of others, thus realizing the fundamental value of the property [5]. Whether the right to personal information can be recognized as a civil right, we must first analyze whether it conforms to the essential attributes of civil rights. Personal information is owned by natural persons, and natural persons can autonomously control and dominate within a specific range and can disclose their information or use it commercially. In order to realize its interests, it reflects the right of natural persons to independently decide how to use personal information, and it is a manifestation of the free development of the personal freedom of the subject of personal information within a certain range [6]. Furthermore, when personal information is disturbed, the right holder can request the counterparty to variation and delete it or request the state agency for compulsory protection, which demonstrates the personal dignity of the natural person. The control and domination of personal information by natural persons also reflect the free exercise of personality power within a certain range [7]. In other words, the right to personal information has already demonstrated a positive willpower, that is, the willpower of self-determination; so, it is a civil right. The theoretical significance of this thesis is to clarify the legal and power attributes of personal information right from the perspective of private law through the specific sorting and analysis of domestic and foreign theories. The location and choice of personal information legislation are determined by the legal attribute of personal information right and the attribution of power attribute. This paper will conduct in-depth research on this theoretical issue and use neural network technology to analyze the rationality of the attribute of personal information right. Therefore, accurately judging its legal attributes is the actual problem of this paper. Article 111 of the General Principles of Civil Law has made relevant rules for the protection of personal information. Therefore, before formulating systematic and comprehensive relevant laws and regulations, defining its attributes is the first step. For the issues to be discussed, more reasonable laws and regulations can be formulated only by clarifying the nature of their rights. Reference [8] believes that personal data refers to any information that has a relationship with a natural person that can be identified or can be identified. A natural person who can be identified refers to one of a series of factors that can directly participate or indirectly refer to its own identification number and its own unique physical, cultural, spiritual, physiological, economic, and social identification and other factors, one or several people who can confirm its identity.

## 2. Related Work

Due to the development of network technology and the speed of changes in the times, personal information itself has great economic value, and there are continuous cases of personal information infringement. People have begun to pay attention to issues with personal information, and the protection of personal information has been a hot topic in academia in recent years, with experts holding a variety of viewpoints and beliefs. At the same time, reference [9] also has a similar definition of the concept of personal information. It believes that the scope of personal information generally includes a natural person's address, name, ID number, personnel records, and birth date medical records and photos and a series of individual or specific personal information that can be identified individually or compared with other information. It is commonly used in the academic community to refer to whether there is a direct relationship between individuals and personal information and to divide personal information into two categories: sensitive information and nonsensitive information [10]. Furthermore, our country's current national standards, “Guidelines for Personal Information Protection” and “Personal Information Security Specifications,” use approaches such identifying connotations and examples for personal sensitive information. Among them, sensitive personal information, if leaked or modified, will have a negative impact on the subject of personal information related to identity. Compared with domestic research, foreign research on personal information started earlier and has a long time, and the personal information legislative protection system is more comprehensive. Looking at the experiences of various countries, in terms of the current international environment, almost all countries in the world protect personal information. Reference [11] officially published “On the Right to Privacy” in 1890, which triggered discussions on the right to privacy in domestic theoretical circles. Since then, the United States has promulgated a special law on the right to privacy, and personal information has been included in the scope of this law in terms of privacy. Reference [12] believes that with the expansion of personal social interpersonal relationships, personal information plays an increasingly important role in social interaction, the relationship between privacy and social interaction is becoming increasingly close, individuals have the right to privacy so that individuals can control the dissemination of their personal information, and the use of third parties is restricted. In actuality, American law has enlarged the area of protection of the right to privacy, and the information subject can freely use and control the information, according to reference [13], which also defaults to the view that privacy is a property of personal information. Individuals can restrict the scope of information activities within the legal limits, according to reference [4], which is an expression of the right to privacy. In terms of personal information protection, as the economization of personality rights progresses, personal information increasingly represents property interests, and a brand-new right, the right of publicity, has evolved in the theoretical circle. The United States uses the right of privacy and the right of publicity to protect the personal interests and property interests embodied in personal information, respectively. In terms of data protection legislation, the United States adopts a segmented legislative approach. Reference [14] believes that the protection of personal information in the United States mainly relies on industry self-discipline, the protection of personal information is scattered in the laws of various states, and the fragmented and fragmented model cannot effectively protect the personal information of its citizens. Reference [15] believes that a right to be forgotten system should be established in line with national conditions. Reference [16] analyzes from the perspective of protecting personal dignity and personal freedom and believes that the essence of protection of personal information rights in European and American countries is to take it as an independent personality interest and incorporate it into the protection of privacy rights. In Germany, personal information is positioned and protected by law in the protection mode of personality rights. The legal interests protected are general personality interests, and Germany is a typical representative. Reference [17] believes that the “other rights” stipulated in article 823 of the “German Civil Code” do not include the right to personal information, and that personal information that reflects the interests of general personality is essentially a system of general personality rights. Reference [18] in his book “The Munich Commentary on the German Civil Code” believes that the right to personal information belongs to the category of “other rights” stipulated in article 823 of the “German Civil Code” and belongs to a separate right. Reference [19] believes that under the framework of German law, whether the right to personal information belongs to the “other rights” in article 823 of the “German Civil Code” or the general system of personality rights, different views on the attributes of the right to personal information will lead to the same conclusion which is that the right to personal information is an absolute right. In terms of German judicial practice, the 1983 “census case” gave birth to a new concept of rights, namely, “information self-determination,” and the right to personal information began to develop in the direction of constitutional rights. At the same time, the Federal Court, based on the “German Basic Law,” affirmed the important value of the right to personal information in protecting personal dignity and personal freedom. From the perspective of doctrine and precedent, Germany recognizes the right attribute of personal information right as a general personality right and realizes the protection of personal information with the use of “information self-determination right.” By analyzing the status quo of personal information rights at home and abroad, it is determined that its legal attributes are mainly the theory of privacy rights, the theory of general personality rights, the theory of specific personality rights, the theory of property rights, and the theory of dual rights. Extraterritorial law mainly identifies the legal attributes of personal information rights as privacy rights and publicity rights, general personality rights, and basic human rights [20–23]. There is a certain gap between the domestic legal tradition and the foreign legislative environment; so, these theories cannot be used for reference. Considering the development trend of personality rights in the new era, it should be considered that certain personality elements reflect certain property interests.

## 3. Method

Here, it discusses the BP neural network. They evaluate the legal attributes and rights attributes of personal information.

### 3.1. Back Propagation (BP) Neural Network

In this subsection, analyze the definition and characteristics of BP network. They define the structure of BP neural network and also discussing the BPNN algorithm. They examine the deficiencies and applications of BPNN.

#### 3.1.1. Definition and Characteristics of BP Network

In the mid-1980s, different scholars independently discovered and proposed the BP algorithm. In 1986, Rumelhart and McClelland published a book titled “Parallel Distributed Processing: Exploration in the Microstructures of Cognition” that had a significant effect on the BP algorithm's implementation. Later, the development of the BP algorithm benefited in the advancement of neural networks by addressing the multilayer perceptron learning problem. The BPNN, a multilayer feed-forward network for algorithm training based on error back propagation, was established in 1986 by a group of academics led by Rumelhart and McCelland. It is one of the most popular neural network models out there. The forward and backward propagations of error are the two main components of BPNN. A neuron in the input layer receives input signals from the external environment and passes them on to a neighboring one or more hidden layers of neurons in the middle layer, which process the transformed data. The middle layer can be a single hidden layer or a multihidden layer structure, depending on the needs of the input signal changes. Direct transmission of learning to the output neurons takes place in a single-layer neural network. A multihidden layer neural network uses a forward propagation method to learn from the previous hidden layer, and then the output layer sends the processing results to the external world. Back propagation of the mistake occurs if the actual output value does not match the predicted output value. Output errors are used to adjust the weights of each layer in the form of error gradient descent, while the error is reversely communicated to the hidden and the input layers. Network learning is an ongoing process in which weights are continually adjusted in order to propagate information and correct faults in a neural network's hidden and output layers. In order for this process to continue, the operator must either be satisfied with the output error or a certain number of learning cycles have been completed.

The information processing technique of BPNN has the following characteristics:

1. Information distributed storage: the BPNN simulates the characteristics of the human brain to store information on the connection strength between neurons and stores the information on the connection weight and distributes it in the network
2. Parallel processing of information: although the speed of human brain neurons transmitting signals is not as fast as that of computers, the human brain can quickly judge and deal with many problems because of its unique properties, which is unmatched by computers. BPNN simulates the human brain to run parallel processing to improve processing power
3. It is fault-tolerant: the BPNN simulates the automatic repair characteristics of the biological nervous system, and the damage of some neurons does not affect the overall error
4. It has the ability of self-learning, self-organization, and self-adaptation. The BPNN can continuously adjust the weights of each layer to adapt to different external environments during learning or training. Under different learning methods, the BPNN can play different network functions. In addition, after training and learning, the BPNN can remember inventory characteristics like as weight matrices and neuron conversion function coefficients and adjust this memory to the inventory, and it may store the system's information distribution in the weight matrix and these coefficients. Changes in the environment are constantly reflected in inventory characteristics, which aid our inventory analysis. BPNN is the core part of the forward neural network. In fact, in the practical application of artificial neural network (ANN), the application of BPNN accounts for a large part of the ANN model. It fully reflects the best part of ANN

#### 3.1.2. Structure of BP Neural Network

Neural networks with several layers are called BPNNs because of their structure. It has three parts: input layer, hidden layer, and output layer. The concealed layer is separated into a single layer and a multilayer structure. For each layer, weights link each node to the next, and each node has a threshold and transfer function for the output layer. The transfer function of BPNN should be differentiable everywhere.

*Input layer:* the input variable of the BPNN is a variable that has a great influence on the output variable and can be extracted with specific values. In addition, as the input variables of the BPNN, the two must be uncorrelated or the correlation is very small.

*Hidden layer:*extracting and storing internal rules from the sample is what this node is all about. For each hidden layer node, there are numerous weights, and each weight promotes network mapping. Generally speaking, complex nonlinear functions with many fluctuations and large amplitude changes require the network to have more hidden layer nodes to enhance its mapping ability. Whether the number of hidden layer nodes is optimal depends on the following factors:

1. The number of input and output layer nodes
2. The number of training samples
3. The noise in the target output
4. The function to be learned by the neural network or the complexity of the classification problem
5. The structure of the network
6. The activation function adopted by the hidden layer nodes
7. The training algorithm
8. The regularization

*Output layer:* generally speaking, the output volume represents the functional goal of the system to be expressed. Under normal circumstances, the output variable is a numerical value, and the system needs to analyze, compare, and study this numerical value. The selection of output variables is relatively simple, and there can be multiple output variables.

#### 3.1.3. BPNN Algorithm

1. Introduction of the neural network algorithm: in 1974, Werbos first proposed the idea of the BP algorithm. Moreover, some other scholars also proposed the BP algorithm in the same period. However, this algorithm has not received the attention of the theoretical community until Rumelhart et al. began to study again. The BP algorithm mainly uses the LMS learning algorithm, which makes the actual result value infinitely close to the expected result value through the gradient search technology. The learning process of BPNN is a process in which the error is propagated backward, and the weights are constantly revised.  Figure 1 shows the algorithm flow of BPNN

In a multilayer ANN, there are two types of signals that are exchanged. When a first-order digital signal is applied to a second-order digital signal and then to a third-order digital signal, the working signal is formed. Input variables and weights of connections determine this. The error signal is the signal from the output layer to the input layer that reflects the difference between the predicted output and the actual output of the neural network. The forward propagation of the input signal and the reverse propagation of the error signal comprise the BP learning algorithm, an iterative process. Its learning method is as follows. The input signal is sent via the transmission process of the input layer-hidden layer-output layer, and the output signal is created at the output layer port. As long as the signal is being sent forward, the network's weights remain constant; therefore, the activity in any given layer of neurons has no effect on the activity in the layer above it. The error signal is transmitted to back propagation if the intended output is not achieved at the output layer. The error signal is the difference between the network's actual output and its predicted output. The back propagation of the error signal occurs when the signal travels from the output layer to the hidden layer to the input layer. Weights in the network are recalculated during the back propagation of error signals. Weights are constantly adjusted to bring the network's output closer to the desired output.

(2) Although the improved BP algorithm of the neural network algorithm has been widely used, it also has its own limitations and shortcomings, such as slow training speed, easy to fall into the minimum point, and low generalization ability. With the continuous in-depth study of the BP algorithm by experts and scholars, many improvement methods have emerged: adaptive learning rate modification and additional momentum methods, for example. First, the adaptive learning rate adjustment method is introduced. There is an optimal learning rate for each specific link of the neural network; so, there are several different learning rates in different stages of a neural network. In order to change this situation and speed up the convergence process, the method of adaptively changing the learning rate came into being. The network automatically adjusts to different learning rates at different stages of neural network training. The adjustment formula is as follows:
  (1) $$\begin{array}{c} \theta \left(t+1\right)=\left\{\begin{array}{cc} 1.15\theta \left(t\right) & E\left(t+1\right)<E\left(t\right),\\ 0.75\theta \left(t\right) & E\left(t+1\right)>1.14E\left(t\right)\\ \theta \left(t\right) & \text{others} \end{array}\right., \end{array}$$

where *θ* is the learning rate, which can be automatically adjusted according to the size of the error *E*.

The second is the additional momentum method. When the neural network uses the additional momentum method to modify the weights of the network, the effect of the error on the gradient and the influence of the change trend on the error surface must be considered. If additional momentum is applied, the network is able to avoid getting stuck in local minima and possibly slip through it. The weight adjustment formula with additional momentum factor is

(2) $$\begin{array}{c} \left\{\begin{array}{c} \Delta w_{ij}\left(t+1\right)=\left(1-m_{a}\right)\theta S_{i}O_{j}+m_{a}\Delta w_{ij}\left(t\right),\\ \Delta v_{ij}\left(t+1\right)=\left(1-m_{a}\right)\theta S_{i}+m_{a}\Delta v_{ij}\left(t\right), \end{array}\right. \end{array}$$

where *O*_*j*_ is the input of the *j*-th neuron in the input layer, *S*_*i*_ is the error signal output by the ith neuron, and *m*_*a*_ is the momentum factor, generally around 0.95.

#### 3.1.4. Deficiencies and Applications of BPNN

Although BPNN has been widely used in the field of prediction, it still cannot cover up the defects of neural network more or less.

(1) The learning rate of ordinary BP neural network is fixed, which leads to slow network convergence and long training time. The learning rate is too small so that the training time of BPNN can be too long. We can use varying learning rates or adaptive learning rates to improve BPNN
(2) The BP algorithm can converge the weights to a value that is likely to be a local minimum rather than a global minimum. We can solve this problem with the additional momentum method
(3) The number of layers and nodes of the hidden layer of the neural network can only be determined through experience or through experiments one by one, which will make the BPNN, have great redundancy, and increase the pressure of network learning to a certain extent
(4) The learning and memory of the network are unstable. The neural network cannot memorize the previous weights and thresholds. If the sample data changes, the neural network has to start training again. But better weights for prediction, classification, or vergence can be saved. The main application of BPNN is as follows:
  - Function approximation: train a grid to approximate a function with training samples consisting of input variables and output variables
  - Pattern recognition: using a pending output variable to associate it with an input variable
  - Categorize: categorize the appropriate way of defining the input variables
  - Data compression: to facilitate transmission or storage, the dimension of output variables can be reduced

### 3.2. Legal Attributes and Rights Attributes of Personal Information

Here, defining the concept of the human right to information, they analyze the dispute over personality rights.

#### 3.2.1. The Concept of the Human Right to Information

The connotation of right is the premise of researching the attribute of a right, and the research on the attribute of personal information right needs to start from its concept. “The General Provisions of the Civil Law” promulgated in 2017 used the expression of personal information in civil legislation for the first time and made it the basis and core concept of article 111, but “The General Provisions of the Civil Law” did not further explain this concept. The concept of personal information first appeared in the data protection proposed in the “International Human Rights Conference” convened by the United Nations in 1968. The expressions of each country vary slightly when compared to the regulations of other countries. Personal information is used in Japan, while personal data is used in Germany and the European Union; personal privacy is used in the United States, replacing personal information with privacy. Different cultural and legal tradition backgrounds in different countries lead to different expressions of data protection, and different expressions are only the relationship between essence and appearance; they are the specific manifestations of information. Based on the above considerations, personal information can better reflect the fundamental rights and interests protected by law. The huge rights system of civil law endows citizens with various rights, and each right is generated based on a specific legal relationship generated by a specific behavior. It takes a long period of development to form a specific right and then join the civil law in the rights system. The most important thing to study a right is to explore its inherent legal attributes. Only by grasping the attributes of a right can the right solve the problems encountered in the real society.

#### 3.2.2. Dispute over Personality Rights

*(1) The General Theory of Personality Rights*. Some scholars believe that personal dignity, equality, and freedom can well protect personal information rights under the theory of general personality rights. The specific reasons are as follows: first, with the development of today's social economy, the nature of the identifiability of personal information rights determines as its scope becomes wider and wider, and it is difficult for a specific personality right to effectively protect the increasingly complex and changing personal information rights, while the openness and inclusiveness of general personality rights in the content of rights can be protected in specific personality rights. Secondly, general personality rights can effectively protect the personal dignity and freedom of natural persons. If the right to personal information falls under the category of general personality rights, it can be adequately safeguarded under the current legal system without the need to create new special rights, which would jeopardize the current system's stability. Finally, there are pertinent practice cases to refer to. For example, in “Ren v. Beijing Baidu Netcom Technology Co., Ltd. Dispute on General Personality Rights,” the plaintiff tried to use the general personality right to claim the “right to be forgotten,” but the law of our country did not provide for this right, and the court finally decided that it was not necessary for protection and did not support it.

*(2) The Theory of Specific Personality Rights*. Some scholars hold the view of specific personality rights for the following reasons: first of all, there are many differences between personal information rights and privacy rights in terms of attributes, objects, and protection methods, and traditional methods of protecting privacy rights and traditional legal protection methods cannot continue to be used. It is easy to cause judicial loopholes, resulting in the inability to effectively protect the right to personal information. It is necessary to defend the personal information of natural persons with a new definite personality right that is different from the right to privacy. Secondly, the development of the market makes personal information generate commercial value. Personal information right not only reflects the interests of personality rights but also reflects certain property interests. The right holder can obtain certain economic remuneration by selling, using, and other means, but it should not be considered that personal information right belongs to the scope of property rights, and its essence still belongs to specific personality rights, while economic value is one of the manifestations in the process of social development. Finally, specific personality rights can coexist with property interests. Personality interests and property interests are not an either-or relationship. With the development of society, there will be more civil rights to reflect the emerging new interests, but this does not affect the original positioning of the rights. The nature of specific personality rights can better safeguard personal information rights.

*(3) Privacy Right Theory*. Scholars who hold a privacy point of view are inevitably influenced by the protection of personal information in the United States and believe that first, in the age of information networks, individuals' attitudes towards personal information related to themselves have undergone a significant change. Second, article 2 of the “Tort Liability Law” specifies the legal attitude toward the protection of the right to privacy. As a result, if the right to personal information is linked to the right to privacy, the right to privacy can be utilized to safeguard it directly without the need to invoke the right to privacy in principle or practice. New rights and solutions, without having to seek new legislation, can leverage mature privacy protection models to maintain legal stability. Finally, in my country's judicial practice, for personal information infringement cases, there are cases based on the right of reputation and the right of portrait, but most cases still use the right of privacy as the cause of the case to define the nature of the case, and the right to privacy is more accustomed to use in practice.

*(4) Property Rights Theory*. Scholars arguing for this theory advocate the right attribute of property rights and believe that in the face of the property interests that constantly reflected by personal information, the traditional personality rights model cannot provide a reasonable explanation for this nor can it be fully protected by the use of personality rights. Therefore, the right attribute of the property right provides effective protection for personal information, and the main reasons are as follows: first, property interests are constantly highlighted. With the development of the market and the wide application of big data, the commercial value of personal information exists as a resource. To some extent, mastering personal knowledge entails mastering future market wealth. The property attribute of personal information rights is becoming increasingly important as data analysis may help corporations change product structure and build individualized marketing campaigns for different consumers, among other things. Secondly, the attribute of property right is a supplement to the theory of personality right. Under the personality rights model, personal information is closely integrated with the subject of rights, has a strong dependence, and cannot exist independently of the subject. However, since entering the era of big data, commercial exchanges have made the commercial value reflected in the information continue to highlight, resulting in many criminals illegally using a large amount of personal information. Therefore, for the separation status of personal information, the use of property rights attributes is an extension and supplement to the traditional theory of personality rights. Finally, attributing personal information rights to property rights is more conducive to the protection of rights subjects. Personal information is vulnerable to illegal infringement in the process of collection and use. Protecting personal information rights in a property rights model can effectively provide adequate protection at all stages of personal information circulation.

According to the various theories of different scholars above, and combined with the specific conditions of the country, this paper constructs a personal information right attribute evaluation system suitable for neural network evaluation, as shown in Table 1. By analyzing the right-related characteristics in the attribute of personal information rights, the rationality of the attribute is judged.

## 4. Experiment and Analysis

Here, it analyzes the dataset sources and defines the BP neural network evaluation model construction. They evaluate the contrastive experiment of BP neural network and the improved model.

### 4.1. Dataset Sources

According to the analysis of the legal attributes and rights attributes of personal information rights in Chapter 3, this paper designs relevant questionnaires and collects and extracts the required data through big data technology. There are 180 groups of data collected, of which 150 groups use as the training set, and 30 groups were used as the test set.

### 4.2. BP Neural Network Evaluation Model Construction

#### 4.2.1. Input and Output Layers

The input layer neurons of the BPNN are the attribute indicators of the personal information analyzed in this paper. In the third chapter, 11 attribute indicators of personal information are analyzed. Therefore, we can set the number of neurons in the input layer of the BPNN to 11 and the number of neurons in the output layer to be 1.

#### 4.2.2. Hidden Layer

This paper designs a 3-layer BPNN model consisting of an input layer, a hidden layer, and an output layer. The number of hidden layer nodes can be selected by the following formula:

(3) $$\begin{array}{c} H=\sqrt{m+n}+a, \end{array}$$

where *H* represents the number of hidden layer nodes, *m* represents the number of neurons in the output layer of the neural network, *n* represents the number of neurons in the input layer of the neural network, and *a* represents a constant in the range [1–9, 24].

Then, the number of hidden layer nodes of the BPNN in this paper is in the range of [3–13]; so, the trial and error method is used to determine the specific value. Select the number of nodes to be 4, 6, 8, 10, 12, and 14 to conduct experiments. The experimental results are shown in Figures 2–4. Finally, the number of nodes selected is 8.

### 4.3. Contrastive Experiment of BP Neural Network and the Improved Model

After the structural analysis of the BPNN, through the training of the training samples, the BPNN fully absorbed the fuzzy and complex laws contained in the training samples. Therefore, using the trained BPNN model to simulate the test samples has a relatively high accuracy. The accuracy of the trained BPNN is uncertain. Here, we must pass the test of the test sample to be sure. The main content of this section is to use 30 sets of test samples to test the trained network and observe its prediction results. Some results are shown in Table 2.

From the results in Table 2, it can be found that the improved BPNN model has smaller error, higher accuracy, and better evaluation effect.

## 5. Conclusion

The fundamental difficulties that must be resolved in the creation of personal information protection legislation are the legal qualities and rights attributes of personal information rights, which are also contentious questions among scholars. There are “basic rights theory” and “private law rights theory,” which comprises “property rights theory,” “personality rights theory,” and “privacy rights theory,” among other things. The “basic rights theory” and the “private law rights theory” genuinely entail the problem of where to place personal information rights for protection when deciding between public and private rights. There is no essential contradiction and can coexist at the same time. The right to personal information can and should be a fundamental right of citizens. However, due to the lack of clear provisions on personal information rights in my country's constitution, coupled with the delay of my country's constitutional interpretation system and the imperfect constitutional litigation mechanism, the right to personal information cannot actually become a basic right in my country. The emergence of commercial entities among the infringing entities and the balance of interests between protecting individual rights and the effective flow of information make it possible for them to be protected in a timely and effective manner only if they are regarded as a private law right in legal policies. Even so, the protection of personal information from administrative, criminal, and other fields is still necessary. This paper builds an assessment index based on the legal qualities and rights attributes of personal information rights and presents a neural network-based rationality evaluation approach for the attributes of personal information rights. The completed work is as follows:

1. Focusing on the legal attributes and the rights attributes is discussed in detail. First of all, the different viewpoints of scholars at home and abroad are introduced one by one, and they are analyzed one by one. Then, summarize and analyze many academic viewpoints and put forward the viewpoints of this paper and demonstrate
2. The evaluation index based on the legal attribute and right attribute of personal information right is constructed, and the BPN model structure required in this paper is determined
3. Compare the results obtained by the BPNN model with the results obtained by the improved BPNN model. The results show that the improved BPNN model has smaller error, higher accuracy, and better evaluation effect

## Figures and Tables

**Figure 1:** BP neural network algorithm flow.

**Figure 2:** Training effect when *N* = 4 and *N* = 6.

**Figure 3:** Training effect when *N* = 8 and *N* = 10.

**Figure 4:** Training effect when *N* = 12 and *N* = 14.

**Table 1:** Personal information right attribute assessment system.

First-level indicator	Secondary indicators	Label
General personality rights	Protect human dignity and freedom	X1
	Equal rights of individuals	X2
	Support the right to be forgotten	X3
Specific personality rights	Enjoy personal interests such as privacy and name	X4
	Enjoy personal interests such as life and health	X5
	Enjoy personal benefits such as reputation and honor	X6
Privacy rights	Include an individual's private life	X7
	Use of personal information, such as sale and transfer	X8
	Insulting information reduces social evaluation	X9
Property rights	Personal information has commercial value	X10
	Collect personal information to meet interests	X11

**Table 2:** Comparison of the evaluation results of the two models with the actual results.

Number	1	2	3	4	5	6	7	8
Actual result	0.812	0.658	0.735	0.859	0.882	0.912	0.622	0.698
BP model	0.785	0.672	0.721	0.828	0.852	0.933	0.665	0.660
Improved BP model	0.821	0.659	0.740	0.849	0.895	0.908	0.638	0.705

## Data Availability

The datasets used during the current study are available from the corresponding author on reasonable request.
